# Enhancing capture efficiency of drug-carrier particles in the carotid sinus by utilizing a combination of magnetic fields: A numerical approach

**DOI:** 10.1016/j.heliyon.2024.e36930

**Published:** 2024-08-26

**Authors:** Mahdi Aali, Adel Esmaeili, Hadi Ebrahimi, Artin Azami, Amir Kavoosi, Somayeh Davoodabadi Farahani

**Affiliations:** a Faculty of Engineering, Islamic Azad University, Central Tehran Branch, 1955847781, Tehran, Iran; b Faculty of Engineering, Arak University, 38156879, Arak, Iran; c Faculty of Mechanical Engineering, Islamic Azad University Khomeinishahr Branch, 8418148499, Isfahan, Iran; d Department of Mechanical Engineering, University of Kurdistan, 416, Sanandaj, Iran; e Department of Mechanical Engineering, K. N. Toosi University of Technology, 19697 64499, Tehran, Iran; f School of Mechanical Engineering, Arak University of Technology, 38181-41167 Arak, Iran

**Keywords:** Drug delivery, Nanoparticle, Carotid artery stenosis, Magnetic drug targeting, Two-phase model, Capture efficiency

## Abstract

Magnetic drug targeting is a relatively new method to treat vascular occlusion in different body parts. However, the effectiveness of this method can be affected due to the severity and location of the occlusion. This can lead to the injection of high dosages of drugs, which can cause serious side effects due to the deposition of drugs in unwanted parts. To mitigate these effects, this study investigates the potential of a guiding magnetic field in enhancing drug absorption for vascular occlusion treatment. The method relies on guiding magnetic nanoparticles (NPs) loaded with drugs toward the occlusion site using two external magnetic fields. Blood flow was modeled as non-Newtonian, considering shear-rate-dependent viscosity and unsteady at the inlet. To test this idea, a computational fluid dynamic (CFD) coupled with a discrete phase model (DPM) approach has been employed to simulate drug delivery in three-vessel structures with varying degrees of occlusion (45 %, 60 %, and 90 %). To avoid the escape of drug carriers, a secondary magnetic field was applied at the bifurcation point to direct the NPs to the site of blockage where the primary magnetic field acts. Then, the states with or without a guiding source at the bifurcation site are compared based on the capture efficiency of each structure. The simulation demonstrated a significant increase in NP capture at the target site, ranging from 2 % to 15 %, depending on the NP size. However, the severity of occlusion substantially impacted the secondary magnetic field's effectiveness. In the 90 % occlusion scenario, the method's efficiency decreased significantly from 26 % to 16 % for NP sizes exceeding 1.5μm. This study highlights the potential of guiding magnetic fields in improving drug delivery to target sites in vascular occlusion.

**Table:** Nomenclature

u	Velocity in x-direction (m/s)	*Subscripts*	
v	Velocity in y-direction (m/s)	p	Particle
w	Velocity in z-direction (m/s)	l	Zero shear rate limit
V	Absolute Velocity (m/s)	∞	Infinite shear rate limit
t	Time (s)	0	ambient
P	Pressure (Pa)	sat	Saturation
S	Component of the magnetic field in each direction	m	Magnetic
n	Number of particles, Power Index	D	Drag Force
F	The magnetization force	f	flow
M	magnetization ($A.m^{-1}$)	in	injected
H	magnetic field intensity ($A.m^{-1}$)	z	z-direction
m	Mass (kg)	y	y-direction
Re	Reynolds number	x	x-direction
r	Radius (m)		
			
*Greek letters*			
$\dot{\gamma }$	Effective shear rate ($s^{-1}$)		
λ	Relaxation time constant		
χ	magnetic susceptibility		
τ	relaxation time (s)		
ρ	Density ($kg.m^{-3}$)		
η	Capture Efficiency		
μ	Viscosity ($N.s.m^{-2}$)		

## 1 Introduction

Cardiovascular diseases remain a leading cause of mortality, claiming the lives of numerous middle-aged and elderly individuals every year. As a result, physicians and researchers in this field constantly encounter challenges in determining the most effective treatments. Many conventional methods, such as radiotherapy, chemotherapy, and surgery, are invasive and carry toxic risks, leading to irreversible consequences, including bone marrow ailments, infection, mucositis, and diarrhea. Consequently, there is a pressing need for safer and low-side-effect treatment alternatives. Researchers have worked on various topics in the last few years, including tissue regeneration and cancer therapy. However, significant progress has been made in drug delivery techniques to precisely target coronary artery diseases and the respiratory system, thereby transforming the aspiration of treating multiple diseases into a reality [[1], [2], [3]]. Numerous drug delivery systems have experienced substantial advancements due to increased utilization and the provision of novel tools by experts [4]. Basically, specialists in this field have focused on improving drug delivery efficiency through active and passive methods. Accordingly, limiting factors have also steered research into more specialized areas. For example, reducing the side effects of high drug doses or the accumulation of nanoparticles at the site of the disease can be highly dangerous [5]. Hence, many nanoparticles with different magnetic properties have been evaluated and tested in recent decades to determine their effectiveness in a magnetic field. In this context, considerable efforts have been made to achieve the highest therapeutic efficiency with the lowest possible injection of nanoparticles [6]. Therefore, a review of research conducted in the past three decades based on experimental and numerical study has been carried out based on various researchers' methodologies and objectives.

Utilizing nanoparticles with various sizes is a crucial factor in enhancing the efficiency of the magnetic drug targeting technique. The efficiency of the magnetic drug targeting method can be improved significantly by applying a diverse range of nanoparticles with different sizes. Hawork et al. [7] studied the impact of particle size on capture efficiency in a magnetic field, assuming non-Newtonian fluid. Based on the Lagrangian method, the model demonstrates that increasing the particle diameter positively affects efficiency. The deposition rate of nanoparticles in a 4-layer artery wall was analyzed by Manshadi et al. [8], considering the effect of porosity and a magnetic field. They found that larger particle diameters and stronger magnetic fields increased particle retention in the plaque area. Akar et al. [9] found that applying a magnetic field to a flow containing nanoparticles in a 90-degree bend increases the mass fraction of nanoparticles in each cell, improving their absorption in the area where the magnetic field is applied. Mohammadpour et al. [10] examined the influence of field intensity and particle diameter on a structure resembling the carotid artery. Their Observations revealed these factors could hinder particle attraction in the occlusion area. Boghi et al. [11] investigated how changing the position and direction of the magnetic field affects the attraction of nanoparticles of different sizes. The coeliac trunk's actual structure was utilized in their study.

Researchers have extensively studied the application of magnetic drug targeting in treating respiratory system-related diseases. It has been observed by Pourmehran et al. [12,13] that an increase in magnetic field intensity leads to enhanced drug deposition in target areas, specifically with fields of B ≤ 1. Gash et al. [14] examined how changing the position of a magnetic field affects particle deposition. Factors such as sleep, rest, and body position were included in their study. Their findings indicated that nanoparticles with larger diameters had better efficacy in weak fields. According to Damoz et al. [15], superparamagnetic iron oxide nanoparticles may have advantages over other types in certain scenarios. In their research, Inthavong et al. [16] focused on analyzing micron particle deposition in laminar pipe bend flows, considering various pipe geometry combinations and flow conditions. In their work, the deposition efficiency is correlated with the particle Stokes number, with a proposed arctan function as a unifying correlation for micron particle deposition in 90-degree bends. Rahimi-Gorji et al. [17] investigated the impact of various factors on the spatial distribution of intraperitoneal (IP) aerosolized anticancer drugs for treating peritoneal metastases. They used computational fluid dynamics (CFD) modeling and experiments to study how droplet size, liquid flow rate, viscosity, and an electrostatic field affect aerosol homogeneity. Mortezaei et al. [18] recognized the importance of accounting for the complexity of the respiratory system in CT scan-based modeling, leading them to utilize fluid-structure interaction (FSI). FSI analysis has also been studied by scientists such as Ebrahimi et al. [19], who investigated its effect on drug capture in abdominal aortic aneurysm (AAA) and wall shear stress. In their study, an optimal amount of drug carriers for the treatment of AAA-related diseases was achieved. Fe3O4@UiO particles were utilized by Rangbar et al. [20] to assess the efficiency of a drug delivery method for COVID-19 patients with the usage of a magnetic field. Due to the reduction in the number of particles, the toxicity caused by this method decreased significantly.

In recent years, magnetic drug targeting has been widely studied for treating carotid artery diseases and enhancing therapy efficiency. Larrimi et al. [21] investigated the effect of an increase in the number of drug carrier nanoparticles entering the external branch of the carotid artery. They demonstrated that the use of a magnetic field close to the external branch can increase particle capture. Hewlin et al. [22] examined factors such as particle capture efficiency, Brownian motion, and change in drug injecting sites using a multi-physics computational model with B = 2T, 4T, 6T, and 8T magnetic fields. Sudagar et al. [23] studied the effect of changing the direction of the magnetic field on particle capture efficiency and found that nanoparticles are more likely to be captured when the field is aligned with the y-axis. By applying the CFD method, Nagargoje et al. [24] studied the flow behavior around the bifurcation of the common carotid and proved that the best location for plaque accumulation is in the sinus section because of vorticities. AliShiri et al. [25] investigated the effect of ultrasonic and magnetic fields on the uptake of drug-coated microbubbles and particles and found that a magnetic field placed in an appropriate location can have a better impact than an ultrasonic field. They discovered that an appropriately placed magnetic field could be more effective than an ultrasonic field. Hossain et al. [26] studied the behavior of blood flow-containing Nanocarriers in preventing strokes due to blockage in the carotid artery and observed some important changes in flow behavior with the manifestation of a magnetic source. Teimouri et al. [27] examined the effect of plaque geometry on nanoparticle deposition. Sulttan et al. [28] developed a mathematical model to predict drug particle trajectories of anticancer dasatinib magnetic nano micelles and found that injection site, particle diameter, and magnetic field intensity have a significant impact on capture efficiency. Schollenberger et al. [29] used MRI scans to improve treatment for carotid artery stenosis and investigated flow behavior in the carotid artery using CFD. They found significant differences in stroke risk based on the degree of blockage and blood pressure differences between patients.

Many advanced methods have been used to improve the treatment percentage of patients and the effectiveness of drug carriers' capture efficiency in disease-affected areas and prevent the side effects of high drug doses as much as possible. One area that has been specifically investigated is magnetic drug delivery to the Internal carotid artery (ICA), which plays a critical role in the occurrence of brain strokes. Several studies have concentrated on investigating how magnetic fields can improve the capture of drug carriers at stenosis sites. These studies have examined factors like nanoparticle size and magnetic field intensity. In addition, changes in the injection site and the wall shear stress have been extensively studied. However, a critical problem in this field is preventing the escape of drug carriers that exit from the External branch in case of ICA blockage. A small percentage of previous research has focused on optimizing the magnetic therapy method by reducing the drug carriers' injected dose. This can accelerate the recovery of patients with cardiovascular diseases and prevent side effects resulting from drug dispersion in the body. Therefore, improving the control and guidance of drug carriers is an issue that has not been specifically examined in detail. Based on this, numerical evaluation of this idea can be a reliable, economical, and rapid option that can better demonstrate the effectiveness of this method before conducting experimental studies.

This article aims to use a guiding magnetic field applied at the carotid artery's bifurcation site to prevent drug carriers' escape into the external branch. Using the computational fluid dynamics (CFD) in the Lagrangian framework, the Discrete Phase Method (DPM) is used to depict the Nanocarrier's trajectories. By establishing two magnetic fields produced by wires carrying current, one positioned at the branching point and the other at the plaque site, particles are directed toward the desired location. First, this model is validated using one of the credible studies [9]. Then, by considering three structures with different occlusions (45, 60, and 90 %), and applying a combination of two magnetic fields, besides examining the efficiency of this method in improving nanoparticle deposition efficiency, dependent parameters such as the velocity and recirculating flows will also be investigated.

## 2 Methodology

### 2.1 Geometry

The carotid artery comprises the most vital blood vessels that supply the neck, face, and brain. Each branch of the common carotid arteries bifurcates into two parts; The internal carotid artery (ICA) carries blood to the brain, while the external carotid artery (ECA) is responsible for blood supply to the organs of the face and neck [30]. This study is based on a realistic model [30] and focuses on various degrees of arterial stenosis at 45 %, 60 %, and 90 % in the ICA. A Cartesian coordinate system is also utilized to evaluate geometric parameters [31]. The geometry of the carotid artery, along with the location of the stenosis and important boundaries, is demonstrated in Fig. 1, one of the three occluded structures studied in this research, drawn based on actual dimensions [32,33]. Stenosis in the internal carotid artery is simulated using models where it has occurred near the bifurcation place at the Carotid sinus.

**Fig. 1:** The geometry, dimensions, boundaries of the carotid artery, and the location of the blockage in the Carotid sinus.

### 2.2 Governing equations

In Fig. 1, blood flow as the working fluid is characterized as viscous, unsteady, incompressible, laminar, and three-dimensional. Due to the blood suspension with drug-carrying nanoparticles, the blood flow is also assumed to be non-Newtonian and bio-magnetic. Therefore, the Carreau equation has been employed to determine the viscose behavior of blood as a non-Newtonian fluid [[34], [35]]. This study utilized the conservation of momentum and continuity equations from the Cartesian system to simulate the flow behavior in the presence of drug carriers and magnetic fields.

For the continuity, it can be expressed as equation (1):

(1) $$\frac{\partial u}{\partial x}+\frac{\partial v}{\partial y}+\frac{\partial w}{\partial z}=0$$

In addition, the Navier-Stokes equations for incompressible flow ${\nabla .u}_{f}$ = 0, considering the relevant terms, can be expressed in an unsteady by equation (2):

(2) $$\rho \left(\frac{\partial u}{\partial t}+u\nabla .u\right)=-\nabla p+\mu \nabla^{2}u+S_{p}$$

In this equation, a coupling between particles and blood flow is established based on the term $S_{p}$ which can be defined as equation (3):

(3) $$S_{p}=n\bar{\left\langle \rho_{p}V_{p}\left(\frac{du_{p}}{dt}\right)\right\rangle }$$

In this equation, in addition to accounting for the particle characteristics denoted by the suffix p and the particle's instantaneous acceleration in the direction of motion, the volume of each computational cell has also been included [[36], [37], [38]].

To investigate non-Newtonian behavior, the viscosity model of Carreau has been used as mentioned, which is presented as follows [34];

(4) $$\mu =\mu_{\infty }+\left(\mu_{l}-\mu_{\infty }\right){\left[1+{\left(\lambda \dot{\gamma }\right)}^{2}\right]}^{\frac{n-1}{2}}$$

In equation (4), $\mu_{l}$ represents viscosity at low values, $\mu_{\infty }$ represents viscosity at high values, and $\dot{\gamma }$ represents the shear rate. It is worth mentioning that the values of n and λ control the fluid behavior between the high and low viscosities. These coefficients are provided in Table 1 [34].

**Table 1:** Coefficient of Carreau model for flow of blood [34].

coefficients	Values	Unit
$\mu_{l}$	0.056	$kg.m^{-1}s^{-1}$
$\mu_{\infty }$	0.00345	$kg.m^{-1}s^{-1}$
λ	3.313	s
**n**	0.3568	–

### 2.3 Nano particles

The trajectory of particles within the blood vessels can be analyzed by considering the inertial forces and forces acting on each particle in its path within an equation. Therefore, it is of utmost importance to meticulously follow the path of each particle individually, which emphasizes the necessity of utilizing the Lagrangian system [[39], [40],^41^]. The Euler-Lagrange model has been employed to trace the nanoparticles and detect their trajectory at any point and time in the flow. This method makes it possible to analyze additional parameters such as the stopping location, particle velocity at each instance, and their behavior upon encountering the magnetic force in the region [42].

The magnetic force generated by the current-carrying wire significantly affects the direction of the particles and is known as the Kelvin force. This force is considered as a volumetric force in the following equation (5) [43]:

(5) $$F_{m}=∭\mu_{0}\;M∙\nabla HdV$$

It is essential to highlight that particles with dimensions within the micron range can align optimally within the magnetic field generated by the wire-conducting current. Furthermore, the magnetization of the particles in that field is approximately in direct proportion to the applied field. It should be pointed out that saturation magnetization is achieved at a magnetic field strength greater than one, at a constant $M_{sat}$ value. Therefore, based on what has been expressed, it can be written as equation (6):

(6) $$M=\left\{ \begin{array}{c} \chi H\;H<M_{sat}/\chi \\ {\;M}_{sat}\hat{H}\;H<M_{sat}/\chi \; \end{array}\right.$$

χ denotes the magnetic susceptibility of particles, which can differ across particle types. Additionally, Ĥ represents the unit vector. Assuming the particles are semi-spherical, the relationship for force can be expressed in a simpler form that can be simplified in the form of equations (7)–(9):

(7) $$F_{m}=\mu_{0}V_{P}M∙\nabla H$$

The forces on a particle can include drag, magnetic, Thermophoretic, Saffman lift, Magnus, Basset, and buoyancy forces. Given the particle diameter, typically exceeding 1 μm, the impact of substantial forces can be disregarded. Furthermore, particles having a diameter smaller than 10 nm are mainly impacted by Brownian forces, therefore these forces can also be neglected.

So the total forces can be expressed as follows:

(8) $$m\frac{d^{2}r}{dt^{2}}=F_{m}+F_{D}$$

In equation (9), $F_{m}$ is the Kelvin force as given in equation (7), and $F_{D}$ is the drag force acting on each particle using the Morsi-Alexander Drag Law, and assuming ${Re}_{p}\equiv \frac{\rho \left|u_{f}-u_{p}\right|D}{\mu }\ll 1$, the following relation for the drag force holds in the present study:

(9) $$F_{D}=3\pi \mu D\left(u_{f}-u_{p}\right),{Re}_{p}\ll 1$$

By combining the two equations and considering $\nabla u\left(t\right)\equiv u_{p}\left(t\right)-u_{f}$:, it can be resulted in equation (10):

(10) $$\frac{d\Delta u\left(t\right)}{dt}=-\frac{\Delta u\left(t\right)}{\tau }+\frac{F_{m}}{m}$$

The relaxation time of the particle is given by equation (11):

(11) $$\tau \equiv \frac{\rho_{p}D^{2}}{18\mu }=\frac{D{Re}_{p}}{18\left|u_{p}-u_{f}\right|}$$

Also, considering equation (8) with Δu=Δu(t=0) and $u_{m}=\frac{F_{m}}{3\pi \mu D}$, it follows that $F_{D}+F_{m}=0$ and, using equation (7) for the particle's velocity [43] it can be expressed as:

(12) $$u_{p}=u_{f}+\frac{F_{m}}{3\pi \mu D}$$

Therefore, in equation (12) the velocity of each particle is calculated at each moment by the sum of the velocity due to the magnetic field and the fluid velocity.

### 2.4 Capture efficiency

The magnetic field created around a current-carrying wire is proportional to the distance from the wire's center. The force experienced by drug particles injected upstream of the flow initially weakens but becomes strong as they approach the bifurcation point of the artery due to a strong magnetic field. This strong magnetic field causes the particles to change direction towards the region of stenosis in the internal carotid artery branch. The force, represented by Formula 7, is introduced to the program as a User Defined Function (UDF). It can produce a maximum magnetic field strength of 2T at the occlusion site. Consequently, while injecting particles using the DPM method, this code calculates the corresponding force that alters the particles' direction based on their distance and relative velocity.

To investigate the precise effect of injecting drug-loaded nanoparticles on therapy and their enhanced effectiveness at the site of stenosis, it is necessary to establish a parameter for measuring the amount of attracted particles at the occlusion site. Hence, the efficiency can be expressed in terms of the injected nanoparticles and the number of particles deposited in target areas around the occlusion site as equation (13) [44]:

(13) $$\eta =\frac{\eta_{trap}}{\eta_{in}}$$

### 2.5 Boundary condition

The distinctive magnetic susceptibility of ${Fe}_{2}O_{3}$ Nanoparticles made them the ideal choice for this study. This is because of the significant amount of iron present in their chemical composition, which is greater than the amount of oxygen, i.e., a 70 % weight ratio of iron to 30 % weight ratio in each mole of the compound. This demonstrates the particles' strong magnetic properties, making them highly effective in delivering drugs to affected areas under a magnetic field [45]. According to the studies [43], this study utilized 10,000 particles with diameters ranging from 0.5 to 2 μm, injecting from t = 0s to t = 0.8s. Table 2 provides an accurate presentation of the compound's details and properties. Also, for better modeling, the shape of these particles is not considered entirely spherical. In this case, we slightly deformed the particles from a spherical state to more irregular shapes using a shape factor of 1.1 to create more realistic results.

**Table 2:** Boundary condition and the properties of injected nanoparticles.

Fluid			Particle (DPM)		
***Boundary condition***					
Inlet	Velocity inlet				
	V = $u_{i}\left(t\right)$		Injection		
Outlet	Pressure Outlet		Escape		
Wall	No-slip Condition		Trap		
***Material***	***Properties***				
	$\rho \left(\text{kg}/m^{3}\right)$	$\mu_{f}\left(\text{kg}/\text{ms}\right)$	$d_{p}\left(\mu m\right)$	χ	$M_{p}\left(\text{kg}\right)$
Blood	1050	0.0035	–		
${Fe}_{2}O_{3}$	6450	–	0.5	3	$4.22\;e^{-12}$
			1		3.38 $e^{-11}$
			1.5		1.14 $e^{-10}$
			2		2.70 $e^{-10}$

Considering that we do not have significant temperature changes, the components related to heat transfer and density are assumed to be constant to define blood fluid characteristics. However, Due to various platelets and globules of different sizes, blood has non-Newtonian viscosity and should be characterized according to valid formulization formulas. Therefore, the Carreau model is used to approximate viscosity effects, ensuring that shear effects are applied to the fluid behavior in the best possible way.

Two magnetic fields also affect these nanoparticles. A current of 100,000 A generates the main field near the stenosis site, leading to a maximum field of B = 2T. Additionally, a variable current based on the diameter of the particles is present in the region where the flow divides into ICA and ECA to deflect the particles towards the occlusion area in ICA. Furthermore, the magnetic field strength in each direction acting on the drug carriers can be calculated from the Cartesian distance from the origin using equation 14–16 [46]:

(14) $$H_{z}\left(z,y\right)=\frac{I}{2\pi }\frac{\left(z-w\right)}{{\left(z-w\right)}^{2}+{\left(y-b\right)}^{2}}$$

(15) $$H_{y}\left(z,y\right)=\frac{I}{2\pi }\frac{\left(y-b\right)}{{\left(z-w\right)}^{2}+{\left(y-b\right)}^{2}}$$

Considering equation (16) as the distance of particles from the magnetic source and the relations related to $H_{z}$ and $H_{y}$ for the intensity of the magnetic field at any location, equation (17) will be valid:

(16) $$r=\sqrt{{\left(z-w\right)}^{2}+{\left(y-b\right)}^{2}}$$

(17) $$H\left(x,y,z\right)=H\left(x,y,z\right)\sqrt{H_{x}^{2}+H_{y}^{2}}=\frac{I}{2\pi }\frac{1}{\sqrt{{\left(z-w\right)}^{2}+{\left(y-b\right)}^{2}}}=\frac{I}{2\pi r}$$

## 3 Numerical method

The equations relating to the continuous and dispersed phase are solved by the Finite Volume Method (FVM). This allows for refining the grid in specific areas, such as boundaries and near vessel walls, in contact with the blood flow compared to other points, which not only increases the accuracy of the solution but also reduces common errors in numerical computation. The accuracy of the solution improves with smaller time steps and converging answers at each step. As a result, when Δt = 0.005s and the simulation is run for 600 steps, the numerical calculations can be completed within a time frame proportional to the CPU's capacity. Fig. 2 shows a comprehensive review of the necessary processes for this numerical simulation.

**Fig. 2:** Flowchart of CFD Simulation and getting results.

The necessary simulations have been successfully executed using the ANSYS Fluent software, which allows for the utilization of multiple computational memories, and the Visual Studio software, enabling us to compile User Define Functions (UDFs) in the Fluent module. This research achieved satisfactory results for each computational time-step by utilizing the Intel(R) Core (TM) i5-5200U CPU @ 2.20GHz and a computational resource of 6GB.

### 3.1 Mesh

This study uses the unstructured grid to solve conservation equations in the computational domain. Additionally, due to the velocity gradients and their impact on fluid behavior, boundary layer meshing is utilized in regions close to the walls with intense gradients. The computational domain must be fine to achieve more accurate particle tracking, and the selected grid should be suitable for fluid behavior and drug particle movements. According to research in this field, due to the complex and multidirectional movements of nanoparticles, it is necessary to consider all possible trajectories, and in applications involving magnetic fields in the presence of magnetic particles, an unstructured tetrahedral mesh can provide a better response [47].

The unstructured grid and boundary layer meshing near the walls are illustrated in Fig. 3.

**Fig. 3:** A detailed view of the boundary layer is presented alongside a 3-D representation of the unstructured mesh.

In the present study, given that the velocity magnitude changes in a pulsatile flow over time and the presence of magnetic nanoparticles in the computational domain, it is necessary to have a mesh with sufficient accuracy. Accordingly, the computational grid should minimize numerical errors and avoid high computational costs. To achieve this, the independence of the computational domain on different values of the elements should be investigated. Fig. 4 shows this process for different grids with various grid elements. Numerical solutions for different structures have been investigated at a line in the bifurcation site. These values were selected as a measure of the independence of the mesh results at t = 0.3. Because of the marginal changes in values beyond 600000, which are in line with grids featuring higher elements, this domain is opted for as the main grid of the project's computational calculations.

**Fig. 4:** A comparison of flow velocity in different mesh numbers on a baseline in the carotid artery bifurcation region.

Then, several grids were created and focused on analyzing the flow velocity in the artery's bifurcation region (Fig. 4). However, as the number of elements increased, we also noted errors resulting from them, especially round-off and truncation errors. Therefore, the first structure that did not significantly affect the results was chosen as the primary representative for numerical solutions and result extraction.

### 3.2 Validation

The study's results by HAVERKORT et al. [43] have been used to validate the present work. Their research examined the deposition percentage of different-sized nanoparticles on a 90-degree bend. Their study employed four magnetic field positions around a 90-degree bend from a spatial perspective. They examined particle capture on the wall, focusing on the location of the electric current-carrying wire near the 90-degree bend. Blood flow was also considered a Newtonian fluid, and the velocity profile at the inlet was considered fully developed. We selected one case from the studied cases to validate our numerical method, analyzed its physics and boundary conditions, and obtained results. Table 3 provides information on the characteristics of magnetic particles and boundary conditions.

**Table 3:** Boundary condition along with the fluid and particle characteristics for the validation of deposition.

Experimental Data for a Typical Run		
Fluid		Particle
Probe. I.D (mm) : 3.95		Material: glass
Flow rate $\left({cm}^{3}/s\right)$ :47.3		
Reynolds number:1000		St: 0.17 ∼ 1.24
Fluid: Air		

To compare the results obtained from the numerical assumptions of the current research and the results of HAVERKORT's study, the graph of the particles' capture efficiency under the influence of a magnetic field in the 90-degree bent tube has been compared. The particle deposition trend after passing through the magnetic field aligns perfectly with the validation graph, confirming the accuracy of our numerical work. Fig. 5(a) illustrates their geometry, structural details, magnetic field, and validation results. The numerical values from the current research and the reference research closely match, as shown in the presented graph. Nevertheless, it is important to note the minor discrepancies among the given values. These negligible differences occur because of the modifications in mesh type, solution algorithm, and convergence criteria and are within an acceptable range of errors.

**Fig. 5:** **(a)**: the capture efficiency of particles versus the change in the nanoparticles' diameter in the research of HAVERKORT et al. compared with the numerical results of the present study. **(b)**: particle deposition on a curved wall in terms of the Stanton number for comparison of the present study and the experimental work of Poui et al. [4].

Also, another simulation has been performed to verify the assumptions made in the current research regarding the type of nanoparticle and its deposition on the artery wall in the absence of a magnetic field. As indicated in Fig. 5, In order to evaluate the behavior of particles outside the bloodstream in a test environment and assess their behavior in the presence of a magnetic field, besides examining fluids, behavioral analysis and particle deposition percentage on the walls need to be investigated. In this way, we have validated our numerical solution through two criteria: validating the particle deposition on a 90-degree curved bend depending on the material type and the efficiency of particle deposition on vessel walls. Thus, utilizing the Poui et al. experiment, it has been demonstrated that in the presence of various types of nanoparticles, the numerical solution can predict the amount of deposition [44]. In their study, different materials, including glass and stainless steel, were considered for injection at the inlet of a 90-degree bend. These materials were subjected to airflow in the order of micrometers and micrograms.

The captured particles in the bend region without magnetic force are ultimately examined and measured. Table 3 provides the boundary conditions and material properties for this validation.

In Fig. 5(a–b), the results of the current research's numerical simulation regarding the deposition of nanoparticles, are provided, along with how they are applied. The accuracy of the experimental research results is satisfactory. This comparison includes the results obtained from glass material and those from stainless steel testing, highlighting the precision of using numerical simulation in predicting the actual behavior of nanoparticles in the absence of a magnetic field.

### 3.3 Results and discussion

This method can potentially enhance the efficiency of drug delivery to vulnerable areas of the body, thereby attracting the attention of physicians to adopt such techniques. Consequently, alongside conventional methods such as radiation therapy and surgery, drug delivery methods can be applied under the influence of magnetic field conductors. However, certain limitations need to be addressed in this context. For instance, precise placement of magnetic fields requires accurate microscopes, and there is also a need for high-tech tools to measure the effectiveness of the treatment concerning the side effects experienced by patients. By overcoming these challenges, magnetic drug delivery could become a valuable addition to the therapeutic arsenal, potentially improving patient outcomes while minimizing adverse effects.

Three structures with different occlusion percentages (45,60, and 90 %) were numerically investigated to analyze the deposition rate of drug-carrying nanoparticles. A pulsatile flow has been introduced at the common carotid inlet to explore the effects of varying flow momentum on the nanoparticle's velocity. This flow, governed by a user-defined function, simulates the blood flow velocity during diastolic and systolic phases, which replaces the actual flow pumping by the heart, presented in Fig. 6(a). Changes in velocity patterns when encountering various stenosis in blood vessels are significant and can affect drug delivery through Nanocarriers in intended areas. Increasing plaque size and, consequently, sudden changes in local velocity and pressure can affect the behavior of the flow and alter its pattern. Fig. 6(b) displays these changes for all three structures with different plaques. The important characteristic of these structures is the drop in blood flow velocity and subsequent increase in particle acceleration due to the narrowed cross-sectional area in the occluded region. For instance, the maximum velocity in the structure with 45 % occlusion is around 0.17 m/s, whereas in the 90 %, this value has quadrupled, which can greatly influence particle capture at this high velocity.

**Fig. 6:** (a): The changes in velocity in the common carotid artery over time at the inlet, (b): The counter of velocity variation among three structures with different occlusions: c (45 %), d (60 %), and e (90 %).

The downstream flow in the ICA is greatly affected by the percentage of stenosis, and the reverse flows in this area are strongly mixed with the main flow. Fig. 7 displays the diagram of blood flow velocity along the x-axis for all three structures. As it is noticeable, the increased degree of occlusion in the ICA leads to a drop in the average velocity in higher percentages. The peak velocity is higher in the structure with 45 % stenosis∼ (0.27 m/s) than in the other two structures (0.25 and 0.05 m/s, respectively). However, the structure with 90 % stenosis showed a significant decrease in velocity along the baseline. After a considerable blockage in this structure, the average velocity along this line has been reduced due to the creation of reverse flows and the subsequent circulating area behind the stenosis, preventing more blood flow from passing.

**Fig. 7:** upstream velocity of the blockage on the given line, based on the occlusion percentage.

#### 3.3.1 Capture efficiency

Using drug-carrying nanoparticles in the body for target areas without a magnetic field cannot have a significant effect and will cause particle dispersion throughout the body. Therefore, particles with various diameters ranging from 0.5 to 2 nm are initially injected. Under the influence of the embedded magnetic field at the plaque site, they are attracted based on their diameters. There is a direct relationship between the deposition of nanoparticles on the targeted point and the applied magnetic force. It's important to note that as the diameter increases, the likelihood of nanoparticle attraction before the plaque site also increases, leading to decreased drug delivery efficiency. Furthermore, some nanoparticles do not reach the intended treatment area as they exit from the carotid artery's external branch.

Hence, the embedded secondary magnetic field can redirect drug carriers to the occlusion site while minimizing nanoparticle deposition in unwanted areas. The main magnetic field acting on the stenosis area now has a greater density of nanoparticles, leading to a significant improvement in drug capture efficiency. A comprehensive investigation has been conducted into the effects of this method.

#### 3.3.2 The minimum required electric current

To create a sufficient magnetic field that can deflect nanoparticles from the external branch towards the ICA, it should be proportional to the diameter of the particles because the force required to direct particles with a diameter of 2 μm is much less than the amount needed for a particle with a diameter of 0.5 μm. The Kelvin force, according to equation (8), is defined as the force applied to the volume of the particles, indicating that $F_{m}\;∼D^{3}$. Therefore, Fig. 8 shows the required electric current to create this field for the spectrum of particle diameters used in this study. It indicates a curved relationship between the minimum necessary electric current for the direction of particles and their size. This required current can be shown as a power function:

$$I_{L}=0.8528D^{-1.254}$$

**Fig. 8:** Minimum electric current required to deflect particles of various sizes in micrometers towards the ICA.

Fig. 9 also shows the contour of changes in magnetic force on nanoparticles and the area where they had their domination. The first-place magnetic particles effectively experience a serious change in their direction is in the proximity of the magnetic field, acting in a region at the bifurcation area, Fig. 9(b). After directing the particles to the occlusion region, the main field Fig. 10(a) attracts nanoparticles with higher density than when the secondary field is not applied.

**Fig. 9:** The distribution of Calvin force in sections of the carotid artery where a magnetic field is applied, a) intensity of the magnetic field in the occlusion site, b) intensity of the magnetic field in the bifurcation.

Table 4 illustrates the capture efficiency of injected nanoparticles under single-field and double-field conditions for various occlusions, depending on nanoparticle size. The criterion for evaluating the efficiency is the deposition of drug carriers at the site of stenosis, which has been detailed for both double-field and single-field conditions in each structure. Increasing the particle diameter has positively improved efficiency, but for better analysis, their graphs should be examined separately to analyze trends. Also, when nanoparticles of various sizes cause 90 % occlusion, there is a noticeable decrease in the structure's efficiency, which we will discuss in detail.

**Table 4:** The efficiency of nanoparticle used in various vascular occlusions with single and double magnetic fields.

Internal Carotid Stenosis (%)						
Particle diameter (μm)	45		60		90	
	CE-1 Field (%)	CE-2 Field (%)	CE-1 Field (%)	CE-2 Field (%)	CE-1 Field (%)	CE-2 Field (%)
**0.5**	9.3	11.6	13.4	14.3	7.6	10.7
**0.75**	13	17	16.6	21.5	9.8	15
**1**	15.5	21.8	19.8	28.6	11.9	19.2
**1.25**	17.3	25.5	23.8	34.4	13.8	23.5
**1.5**	18.3	28.6	27.8	40.2	14.9	25.9
**1.75**	18.8	30.6	29.7	42.7	15.2	22.9
**2**	18.9	32.1	31.5	45.1	14.9	16.1

In Fig. 10(a–c), graphs have been plotted to understand better the relationship between the presented values of nanoparticle capture efficiency and compare the performance of separate structures for each degree of blockage. In Fig. 10(a), where the plaque degree is lower (45 %), the deposition efficiency in both scenarios follows an increasing trend. However, using a deflector field in the bifurcation section has improved this value, leading to a significant increase in efficiency with the increase in particle diameter. In this structure, the efficiency in smaller particles has resulted in approximately 2 % growth in efficiency when the magnetic deflector is applied. On the other hand, an improvement of roughly 14 % can be noted in larger sizes, proving the point that capture efficiency at the target site has a direct relationship with the increase in particle size.

**Fig. 10:** Comparison of particle capture efficiency at the blockage site based on single and double magnetic field: a: 45 %, b: 60 %, c: 90 %.

The presence of a secondary magnetic field that guides particles toward the ICA positively impacted particle capture efficiency in all three cases. However, variations in the patterns were observed. On the other hand, in the 90 % blockage scenario (Fig. 10(c)), efficiency significantly dropped when exposed to a double magnetic field. The decrease was also observed when the particle diameter increased from 1.5 μm in the single-field structure. It is crucial to thoroughly examine the consequences of flow forces and reverse flow in this context, as they possess enough strength to surpass magnetic field force and lead to a notable deflection in particle deposition. Valuable information on flow behavior and its impact on nanoparticle movement can be obtained from the flow streamlines passing through the carotid artery and occlusion site in Fig. 11. When the blockage reaches 45 %, reverse flows and their visible center are observed in Fig. 11(a), causing changes in the fluid path in the internal carotid. As the blockage increases to 60 %, the reverse flow moves back with its core positioned farther away than the 45 % occlusion.

**Fig. 11:** The middle surface provides a 2-D view, illustrating the formation of reverse streams in the region leading to the stenosis site: a) 45 %, b) 60 %, c) 90 %.

In the 60 % blockage state (Fig. 11(b)), the particle capture efficiency exceeded that of the 45 % blockage state. This can because of the point that, by combining reverse flow with the main flow and placing the circulating core in the center, where maximum blood velocity occurs, flow energy is significantly diminished. As a result, because of the direct relationship between magnetization and the force for particle deflection outlined in Equation (13), particles tended to be directed more by the deflector field when 60 % blockage occurred. Hence, they enter the target area with less required force and are easily captured by the main magnetic field at the plaque site.

As the blockage in the artery reaches 90 % and the plaque becomes considerably large (Fig. 11(c)), it creates a vortex field that covers the entire artery width. Therefore, by creating a reverse-flow domain that acts as a huge barrier, many nanoparticles are diverted away from their intended destination back to the bifurcation site.

### 3.4 Capture or escape in peripheral sites

After investigating the impact of a deflector field on nanoparticle deposition efficiency at the stenosis site, examining the capture rate at other sites is crucial. The aim is to assess the increase in efficiency resulting from the deflector field, compared to the nanoparticle output from the ECA when only the main field is employed. Determining the connection between the reduction in nanoparticle output from the ECA and the efficiency improvement following the second field's application is essential. The relationship, which has been investigated in three different occluded structures, is depicted in the diagrams presented in Fig. 12. In the first two structures (45 and 60 %), as the particle diameter increases, there is a direct relationship between the reduction in the output of nanoparticles and the increase in efficiency at the stenosis site. This is because smaller particles are less affected by the magnetic field force. Still, efficiency improves with increased diameter and greater magnetic field susceptibility. At the same time, the output from the ECA decreases due to the influence of this dominant field at the bifurcation site. However, for the structure with 90 % stenosis, as discussed earlier, this relationship has resulted in a decreasing trend on both diagrams after the diameter of 1.5.

**Fig. 12:** Comparing the output of nanoparticles in the external carotid artery in a single field versus enhanced efficiency with a second field; a) 45 % occlusion, b) 60 % occlusion, c) 90 % occlusion.

The attraction of particles to peripheral walls upstream of the blockage occurs because of factors such as the guiding field's influence and the formation of recirculating flows. In Fig. 13, particles are deposited at undesired points and upstream areas before the 90 % blockage. More than 70 percent of particles larger than 1.5 μm have been captured in a different neighborhood from the blockage.

**Fig. 13:** The amount of particle capture at points at the unwanted points in the structure with 90 % obstruction.

Fig. 14 displays this relationship through the nanoparticle trajectories, Fig. 14(a) and the contour of streamlines, Fig. 14 (b). The accumulation of particles is considerable at the end of the vortex region (tip of streamlines) due to the drop in velocity, change in direction, and flow circulation behind the 90 % blockage site. The simultaneous effect of the vortex region and the second field's magnetic force suggests that the inferior point, shown in Fig. 14(a), captures approximately 80 % of nanoparticles.

**Fig. 14:** The Location of peripheral capture on the bifurcation site, **a**: The accumulation of nanoparticles near the junction, **b**: The formation of reverse flow.

The performance of the double-field method has been analyzed sufficiently, so in this section, the direction of the ${Fe}_{2}O_{3}$ particles, considering their velocities is shown in the form of particle trajectory contours in Fig. 15. The injection of nanoparticles into the upstream flow (common carotid) and their movement towards the ICA due to the deflector field have been demonstrated. When particles are injected into the fully developed flow, they take on this shape due to the Parabolic flow motion. These snapshots illustrate the path of drug carriers at different times and the function of the magnetic barrier field in the bifurcation region, preventing particles from entering the external carotid artery. This field is displayed in terms of force per cubic meter.

**Fig. 15:** The snapshots of injected nanoparticles into the common carotid and their paths.

## 4 Conclusion

In the current project, we employ the finite element method to analyze three structures with different occlusions, providing a reliable approximation of the real geometry for various parameters. Key aspects have been thoroughly investigated, including particle capture efficiency, blood flow circulation's impact on nanoparticle deposition and movement, and peripheral particle capture. In this regard, a spectrum of nanoparticles (10,000) ranging from 0.5 to 2 μm were injected to act in a domain with a combination of magnetic fields, including the main field ($10^{5}A$) at the blockage site and the directing one, acting near the ECA. Three structures with different blockage percentages in the sinus region have been considered. Reliable results on the effectiveness of the CFD method have been obtained by assuming the main forces acting on drug-carrying nanoparticles. It improves nanoparticle capture and reduces the need for extra injection and associated drug toxicity risks. Several simplifications have been considered, such as ignoring forces that have a minimal impact on nanoscale drug carriers. Moreover, this study overlooks the viscoelastic behavior of the artery wall and its effect on drag force. Nevertheless, these factors are unlikely to impact this method's efficiency in the blockage area. In summary, these results can be categorized as:

• Changing the direction of drug-carrying nanoparticles through a guiding magnetic field at the bifurcation area positively enhances the capture efficiency at the target site. In this regard, on average, in structures with 45 %, 60 %, and 90 % occlusion, the improvement of the efficiencies is 23 %, 32.4 %, and 19 %, respectively.
• The efficiency relies heavily on the degree of blockage in the internal carotid artery, which hinders the delivery of nanoparticles to the target site for treatment due to the formation of reverse flows caused by the localized blockage. In the structure with 90 % blockage, 80 % of Nanocarriers failed to be captured by the target site, leading to attraction in unwanted walls.
• Increasing the particle diameter also increases their deposition on the stenosis region. Only in 90 % of blockage when the particle diameter exceeds 1.5 μm does a significant reduction in capture efficiency occur. With an efficiency of 16 % in the attraction of 2-μm drug carriers, it falls below the average (19 %).
• The vortex region decreases the particles' velocity and reduces the minimum force required to deflect them. Consequently, upon detaching from the flow path, these particles reach the bifurcation site at a low speed and get attracted by unwanted areas.
• The deflection of particles ranging from 0.5 to 2 μm requires a minimum force that is highly nonlinear and exponential. Therefore, altering the trajectory of smaller particles requires a stronger electric field.
• As the blockage level within the internal branch rises, there is a significant drop in the average flow velocity in the artery. This drop in velocity is related directly to the recirculating flows, which cause the dissipation of a considerable amount of blood flow energy within this branch. in this regard, peak velocity is related to the structure with lower blockage, which is 45 %, with a peak velocity of 0.27 m/s.

## CRediT authorship contribution statement

**Mahdi Aali:** Writing – review & editing, Writing – original draft, Validation, Supervision, Software, Resources, Methodology, Data curation, Conceptualization. **Adel Esmaeili:** Writing – review & editing, Software, Methodology, Data curation. **Hadi Ebrahimi:** Software. **Artin Azami:** Validation, Formal analysis. **Amir Kavoosi:** Writing – review & editing, Validation, Formal analysis. **Somayeh Davoodabadi Farahani:** Writing – review & editing, Supervision, Project administration, Formal analysis, Data curation.

## Declaration of competing interest

The authors state they do not have any financial conflicts of interest or personal relationships that could have potentially influenced the findings in this paper.
